# Determination of the Proportion of Total Soil Extracellular Acid Phosphomonoesterase (E.C. 3.1.3.2) Activity Represented by Roots in the Soil of Different Forest Ecosystems

**DOI:** 10.1100/2012/250805

**Published:** 2012-06-04

**Authors:** Klement Rejsek, Valerie Vranova, Pavel Formanek

**Affiliations:** Department of Geology and Soil Science, Mendel University in Brno, Zemedelska 3, 613 00, Brno, Czech Republic

## Abstract

The aim of this study is to present a new method for determining the root-derived extracellular acid phosphomonoesterase (EAPM) activity fraction within the total EAPM activity of soil. EAPM activity was determined for roots, organic and mineral soil. Samples were collected using paired PVC cylinders, inserted to a depth of 15 cm, within seven selected forest stands. Root-derived EAPM formed between 4 and18% of the total EAPM activity of soil from forests of differing maturity. A new approach, presented in this work, enables separation of root-derived EAPM activity from total soil EAPM. Separation of root-derived EAPM from soil provides a better understanding of its role in P-cycling in terrestrial ecosystems. The method presented in this work is a first step towards the separation of root- and microbe-derived EAPM in soils, which are thought to possess different kinetic properties and different sensitivity to environmental change.

## 1. Introduction

Extracellular acid phosphomonoesterase (EAPM) (orthophosphoric monoester phosphohydrolase, E.C. 3.1.3.2) plays an important role in the mineralization of soil organic phosphorus in a range of terrestrial ecosystems [1, 2]. This enzyme may be produced in soil by microorganisms including bacteria, protozoa, and mycorrhizal or saprophytic fungi and by plant roots [3–5]. Root-derived EAPM is bound onto root surfaces or released to external media as a part of the root exudates [6].

Different ecosystems are thought to have either plant- or microbe-derived EAPM prevailing in soil [7, 8]. Nevertheless, there were no available data indicating the significance of plant roots *versus* soil microorganisms in the production of EAPM and thus their relative importance for P-cycling. EAPM from roots is known to possess different kinetic properties and sensitivity to other factors of environment compared to that derived from microorganisms [9]. Consequently, these two fractions of total soil EAPM may respond differently to climate change and other environmental perturbations [6].

Separation of plant root- and microbe-derived EAPM in soil is difficult. Hence, we have developed a new approach, focusing on the activity of root-derived EAPM as a part of the total EAPM activity of soil in different forest ecosystems.

## 2. Material and Methods

### 2.1. Site and Soil Sampling

In total, seven forest stands were selected for this study. These included young (19 years) and old (207 years) beech (*Fagus sylvatica* L.) stands (480 m asl, N 49°16′54′′, E 16°37′52′′), young (33 years, oak 60%, hornbeam 30%, beech 10%) and old (133 years, oak 87%, Douglas fir 6%, beech 4%, and larch 3%) oak (*Quercus robur *L.) stands (460 m asl, N 49°32′16′′, E 16°79′75′′), and young (15 years, spruce 100%), middle-aged (51 years, spruce 68%, larch 32%), and old (94 years, spruce 92%, larch 6%, beech 2%) spruce (*Picea abies* L.) stands (500 m asl, N 49°32′19′′, E 16°78′54′′). Soils within the studied stands were Dystric Luvisol (young beech and old oak), Haplic Cambisol (old beech and young oak), Dystric Cambisol (old spruce), Gleyic Cambisol (young spruce), and Leptic Cambisol (middle aged spruce) [10].

Five pairs of PVC cylinders (15 cm long, 5.9 cm dia) were randomly inserted in every stand; cylinders within the same pair were always inserted side by side, to ensure similarity. After transportation to the laboratory in plastic bags, the litter layer in all cylinders was removed. One cylinder in each pair was used for separation of all the roots, which were washed in tap water and then in demineralized water. The soil from the second cylinder was separated into organic (F + H horizons) and mineral part to ensure consequent determination of EAPM activity of naturally developed soil layers without their artificial mixing together both parts were separately sieved through a 5 mm mesh, homogenised, and weighed.

### 2.2. Root Analysis

All roots from each of the cylinders were incubated, in succinate-borate buffer (pH 4.8) at 37°C for 30 min., with p-nitrophenyl phosphate (p-NPP) as a substrate [11]. The substrate dissolved in succinate-borate buffer was applied in ratio 12 mL per 0.5 g of fresh roots.

### 2.3. Soil Analysis

EAPM was measured separately in organic and mineral soil. Fresh soil (1 g) was incubated, in 12 mL of succinate-borate buffer (pH 4.8) at 37°C for 1 h, with p-NPP as a substrate [11]. EAPM activity was consequently calculated per the total amount of organic and mineral soil of every cylinder (data were pooled together), and, further, EAPM of roots of the same cylinders was added to obtain the total EAPM of the whole cylinder. Results were consequently calculated per 100 cm^2^ of soil surface.

### 2.4. Statistical Treatment

Values are given as means of five replicates with standard errors (SE). Significant differences were calculated using one-way ANOVA plus Fisher's LSD test.

## 3. Results and Discussion

The total soil activity of EAPM, including roots, was significantly (*P* < 0.05) higher in young oak, old oak, and young spruce than that in other forest stands (Figure 1). Significantly (*P* < 0.05), the lowest total EAPM activity was found in the soil from the old beech forest stand. From the total EAPM activity of soil, up to 18% was derived from roots (Figure 2). The proportion of root-derived EAPM was higher for all spruce stands (at average >12%) than for beech or oak stands, due to higher EAPM related to unit fresh root mass (Table 1).

Historically, different approaches have been tested to separate acid phosphomonoesterase activity in soils. These have included separation of the intra- and extracellular APM pool [12–15], assessment of APM in rhizosphere *versus* bulk soil [3, 16, 17] or within particle-size fractions [18–20], soluble *versus* immobilized soil APM fractions [21–24], or phosphatase bonded to humic substances [25]. In addition to these, fractions of APM derived from plant roots have been studied in intact roots, external-root solution (as a part of rhizodeposition), root apoplastic sap, total root, and root segment extracts. Anatomical-physiological studies of surface-bound phosphomonoesterase activity in cross sections of roots and mycorrhizal associations have also been carried out [3, 6, 26–29].

As APM from roots and microorganisms is known to possess different kinetic properties, separation of APM sources in soil components allows us to better understand the response of P-transformation in soil in different conditions. The new approach presented in this work does not enable us to distinguish between root- and microbe-derived EAPM in soil, nor can we determine if the studied forest ecosystems have either plant- or microbe-derived EAPM prevalent in the soil. Nevertheless, the presented approach enables separation of root-derived EAPM activity from EAPM of the soil which may originate from both microorganisms and roots. The results presented in this work showed up to 18% of EAPM in soil to be root-derived when mycorrhizal status of roots was not considered. This work represents a first step in research leading to separation of root- and microbe-derived EAPM in soils.

Origin of phosphomonoesterase was shown to affect its Michaelis-Menten characteristics (*K*_*m*_ and *V*_max⁡_ values) and response to pollutants (e.g., Cu) and other compounds in soil [30, 31]. Also, Gould et al. [9] reported that properties of microbe- and root-derived EAPM were different including their kinetic parameters and temperature sensitivity. Further research is necessary to separate the importance of root- and microbe-derived sources of EAPM in the soils of different ecosystems in order to better understand their importance in P-cycling and to evaluate their sensitivity to climate change and other types of environmental perturbations.

In conclusion, root-derived EAPM forms a lesser part of the total EAPM activity of soils in forest ecosystems. These findings can be generalized for acid forest soils where EAPM is of microbial and root origin. Alkaline soils with dominance of alkaline phosphomonoesterase of microbial origin are hypothesised to have especially plant root-derived EAPM activity; however, it still remains to be experimentally determined.

## Figures and Tables

**Figure 1:** Total soil activity of EAPM, including roots (up to 15 cm depth), from seven forest stands (Mean ± SE). Different letters (in brackets) mark significant differences (*P* < 0.05).

**Figure 2:** Proportion of root-derived EAPM within total soil EAPM up to 15 cm depth (Mean ± SE).

**Table 1:** Total Root Mass and EAPM Activity of Roots in Seven Forest Stands (Mean ± SE). Different Letters Mark Significant Differences (*P* < 0.05).

Forest	g fresh roots	mg p-NP g^−1^ fresh roots h^−1^
Young beech	3.98 ± 0.85^a^	0.27 ± 0.03^a^
Old beech	6.79 ± 1.10^ab^	0.17 ± 0.03^a^
Young oak	7.49 ± 1.27^bc^	0.26 ± 0.02^a^
Old oak	9.77 ± 1.00^cd^	0.27 ± 0.02^a^
Young spruce	4.18 ± 0.52^ae^	1.18 ± 0.10^b^
Middle-aged spruce	6.95 ± 0.86^bde^	0.58 ± 0.08^c^
Old spruce	4.02 ± 1.11^a^	0.81 ± 0.13^d^
